The article "EEG-Based Personality Prediction Using Fast Fourier Transform and DeepLSTM Model" was published in 2021. Journal: Comput Intell Neurosci.

# EEG-Based Personality Prediction Using Fast Fourier Transform and DeepLSTM Model

**DOI:** 10.1155/2021/6524858

**Published:** 2021-09-20

**Authors:** Harshit Bhardwaj, Pradeep Tomar, Aditi Sakalle, Wubshet Ibrahim

**Affiliations:** ^1^CSE Department, Gautam Buddha University, Greater Noida, India; ^2^Department of Mathematics, Ambo University, Ambo, Ethiopia

## Abstract

In this paper, a deep long short term memory (DeepLSTM) network to classify personality traits using the electroencephalogram (EEG) signals is implemented. For this research, the Myers–Briggs Type Indicator (MBTI) model for predicting personality is used. There are four groups in MBTI, and each group consists of two traits versus each other; i.e., out of these two traits, every individual will have one personality trait in them. We have collected EEG data using a single NeuroSky MindWave Mobile 2 dry electrode unit. For data collection, 40 Hindi and English video clips were included in a standard database. All clips provoke various emotions, and data collection is focused on these emotions, as the clips include targeted, inductive scenes of personality. Fifty participants engaged in this research and willingly agreed to provide brain signals. We compared the performance of our deep learning DeepLSTM model with other state-of-the-art-based machine learning classifiers such as artificial neural network (ANN), K-nearest neighbors (KNN), LibSVM, and hybrid genetic programming (HGP). The analysis shows that, for the 10-fold partitioning method, the DeepLSTM model surpasses the other state-of-the-art models and offers a maximum classification accuracy of 96.94%. The proposed DeepLSTM model was also applied to the publicly available ASCERTAIN EEG dataset and showed an improvement over the state-of-the-art methods.

## 1. Introduction

Personality has been developed from different theories, but personality core is a function of individual behavioral differences and experiences affected by an individual's development, such as his/her emotions, social relationships, and life experiences [1]. Personality represents the action style of a person in daily life. There are many theories and personality measurements, but the personality trait measurements have become the most considerable acknowledgment in the scientific community and play an irreplaceable role [2].

There are various ways in which personality prediction can be made. Personality can be identified by filling out questionnaires, also known as self-reported personality assessment. The five-factor personality test [3] and MBTI personality test [4, 5] are its examples. Personality prediction can also be made using social media such as Twitter [6] and Facebook [7] data, but that is not always so accurate because the data can be fake [8–10].

The article "EEG-Based Personality Prediction Using Fast Fourier Transform and DeepLSTM Model" was published in 2021. Journal: Comput Intell Neurosci.

The personality prediction using physiological signals has recently received a lot of interest [11]. The physiological signal allows researchers to have a better understanding of the participant's reactions during the experiment. Recognizing personality from physiological signals [12–14] is more accurate than digital footprints [15, 16] because this approach achieves a higher classification accuracy.

Among the physiological signals, the electroencephalogram (EEG) signals have grown in prominence in recent years and have achieved a higher classification accuracy [17, 18]. The electrical activity produced by neurons in the brain is recorded using EEG, which have been widely utilised to study functional changes in the brain [19, 20].

EEG signals frequency varies from 0.5 Hz to 100 Hz and is grouped into five bands: delta, theta, alpha, beta, and gamma; all the bands have different frequencies [21, 22]. A band of 0.5Hz–50 Hz is used for this paper.

The main contribution of this paper is as follows:

- The newly EEG dataset is created for personality prediction using NeuroSky MindWave Mobile 2 device
- This study proposed a DeepLSTM model for the prediction of personality traits

The remaining paper is structured in the following manner.  Section 2 provides background details.  Section 3 is devoted to the materials and methods used in this study.  Section 4 discusses the proposed personality framework.  Section 5 provides the experimental results.  Section 6 discusses the comparison of the proposed DeepLSTM model with the other state-of-the-art methods.  Section 7 presents the conclusion.

## 2. Background

This section explains the FFT for extraction of the features and is discussed in detail next.

### 2.1. Fast Fourier Transform

The first step in the successful classification [23, 24] of personality traits is to extract important EEG signal features. The popular methods for analyzing EEG data are decomposing signals into various frequency bands, as shown in Figure 1, including delta (0.5 to 4 Hz), theta (4 to 8 Hz), alpha (8 to 12 Hz), beta (12 to 30 Hz), and gamma (30 to 100 Hz). The MindWave can use the onboard chip ThinkGear ASIC Module (TGAM1), with algorithms that reduce the background noise and objects. For a decomposing signal with fast Fourier transform (FFT), the TGAM1 chip has an algorithm. The value is provided to the application program by the TGAM1 chip using the device. Each second data are gathered and processed in the temporal field to identify and correct as much as possible the artifacts and background noise, without the practical usage of NeuroSky's proprietary algorithms, of the original signal. The headset helps us to control meditation and attention features that their eSense technology measures.

The article "EEG-Based Personality Prediction Using Fast Fourier Transform and DeepLSTM Model" was published in 2021. Journal: Comput Intell Neurosci.

## 3. Materials and Methods

This particular section gives details about the pool of participants, details about the device used for experimentation, the details of the dataset used for experimentation, and lastly details about the procedure of experimenting.

### 3.1. Pool of Participants

This study consists of 55 participants. However, five samples have been removed from the final assessment due to dware errors or inappropriate EEG signal artifacts. Therefore, 50 representative samples of 18 to 46 years of age (25 males and 25 females) participated in the study. Forty participants are handed to the right; ten are handed to the left, each with a natural vision. Participants were not allowed 24 hours before the experiment to take tobacco or caffeine.

### 3.2. Device Description

The NeuroSky MindWave mobile 2 device's functionality is to capture brain signals, as seen in Figure 2. The brainwave reading EEG headset is simple to monitor and is cheap. It generates 12-bit (3–100 Hz) raw brainwaves at a 512 Hz rate and generates EEG power spectrums at various frequency and morphology bands. It is used for pairings with a static headset ID. For capturing the dataset, eegId application is used, which has in-build FFT feature extraction technique and ten features are extracted.

### 3.3. Proposed EEG Dataset

Visual content is a reliable means of eliciting affect or emotion [25] in the literature. We created and consolidated a set of 40 movies and series clips for this analysis, which served as elicitation materials for the data collected from subjects. The content of these movie clips includes audio and video elements, allowing students to participate in immersive experience. English language and Indian language (Hindi) film samples with a length of about 2 to 4 minutes were chosen for the process. Each clip in the elicitation material includes content that evokes emotions and personality traits and characters exhibiting a particular personality trait.

All of the chosen movie clips are thought to generate and activate the desired personality trait's characteristic emotions.  Table 1 presents a selection of stimuli dataset clips used to evoke a particular personality trait for EEG data acquisition. The order and selection of clips were randomized to ensure effectiveness.

### 3.4. Publicly Available Dataset

This research also uses the publicly available EEG dataset of personality known as ASCERTAIN dataset [26]. The ASCERTAIN dataset uses the BFF model for personality prediction using EEG signals, which have been collected in laboratory settings from the single-channel EEG device. The recorded information includes frontal lobe activity, level of facial activation, eye-blink rate, and strength. It contains 58 participants' EEG recordings as data, and 36 movie clips were taken. These clips are between 51 and 127 s long. All topics were popular in English, and the students were regular film watchers from Hollywood. The film clips (nine clips per quadrant) are distributed uniformly throughout the visual analog (VA) space. For the recording of physiological signals, different sensors were used in the surveillance of the clips. After watching the clip, each participant was asked to mark the VA scale with a 7-point scale to represent his practical experience. The personality test for the five large dimensions has also been evaluated using a 5-dimensional questionnaire.

The article "EEG-Based Personality Prediction Using Fast Fourier Transform and DeepLSTM Model" was published in 2021. Journal: Comput Intell Neurosci.

## 4. Proposed Personality Prediction Framework Using EEG Signals and DeepLSTM Model

Figure 3 includes the entire framework for personality prediction using EEG signals and the DeepLSTM model. The proposed framework consists of two parts. First is the data collection for personality prediction, and second is the DeepLSTM model for classification of personality traits, and both of these are described next.

### 4.1. Data Collection for Personality Prediction

Data collection is the first step in the research process. This dataset was obtained using an experimental protocol that is well established and easy to follow. The dataset is created to support 50 volunteers (25 men and 25 women) who will be actively involved in the data collection process. Since an individual's personality trait cannot be assessed solely by their current mood or state of mind, the data will be collected three times over five days [27]. The participant was initially relaxed in the data collection process and wore the NeuroSky MindWave mobile 2 headset on their head. Since there are four groups in the MBTI personality traits, each group consists of two traits in verses of each other. There are eight traits, and for each trait, one film clip is shown to the participant. During the training time, the proposed procedure is iterated eight times with one participant. Before each film clip, the participants were given a 20-second starting hint to begin the test, during which they viewed video clips of a targeted personality trait. Following that, each participant signs a consent form, which is then accompanied by keeping a record of their general information such as name, age, and gender at the initial levels for developing the dataset. Single-channel EEG adjustable headband was used to monitor the EEG signals.

The article "EEG-Based Personality Prediction Using Fast Fourier Transform and DeepLSTM Model" was published in 2021. Journal: Comput Intell Neurosci.

After viewing a film clip of one trait, the participants had to fill the self-evaluation form with options “agree,” “neutral,” or “disagree” and have seven questionnaires for each personality trait. These questionnaires are constructed by targeting the characteristics of personality traits. These questionnaires must be answered based on the participants' real feelings instead of their typical emotions or general attitude, which may differ from person to person. Because of that, the answer to those questionnaires may differ. In each clip, a 1-minute buffer is for neutral clip to neutralize the participants' elicited personality traits. After all of the questions for each of the four grouped personality traits have been answered, the questionnaire (which contains seven questions) is evaluated for each participant's traits. The labeling of the EEG signal depends on the output of the questionnaires given by the participant. The final output is evaluated by the following procedure. Let us suppose that the participant has watched the film clip targeting the characteristic of the extraversion trait. After watching the film clip, the participant answered the questionnaires based on the extraversion trait. Suppose the participant selects for the “agree” option in the questionnaire. In that case, we can raise it by value 1. If, for the extraversion questionnaire, the participant chooses the option “disagree,” we raise the counter of the introversion trait (versus trait of extraversion) by one. If the participant opts for the neutral option, we neither increase nor decrease the counter for any trait. Since there are seven extraversion trait questionnaires, the EEG signal labeling depends on the participant's output, and three labeling possibilities exist.

- The EEG signal is labeled as extraversion if the number of “agree” options is more selected than “disagree”
- The EEG signal is labeled as introversion if the number of “disagree” options is more selected than “agree”
- The EEG signal is discarded if the number of “agree” and “disagree” options are equal in number

Similarly, for introversion trait-based questionnaires, the counter for introversion trait is incremented if the participant chooses the “agree” option. If the participant chooses the “disagree” option, the counter for extraversion is incremented. If the participant opts for the neutral option, we do not increase or diminish the counter for that questionnaire of both the traits. The labeling of the EEG signal is done by following the above procedure. Similarly, the remaining personality traits marking is done, and their related EEG signals are labeled. The same experimental procedure is repeated after three days for collecting the data and removing bias.

The article "EEG-Based Personality Prediction Using Fast Fourier Transform and DeepLSTM Model" was published in 2021. Journal: Comput Intell Neurosci.

At the end of each trait's evaluation process, the dataset's maximum counter value is labeled. To label the EEG signals, this marking scheme is taken as the reference. The study's testing data were obtained using just four video clips, targeting one personality trait from each group.

The experiment will be performed using four machine learning algorithms, ANN, KNN, LibSVM, and HGP, including our proposed DeepLSTM classifier. The survey and review of results for the recorded EEG signal dataset using the described machine learning algorithms will provide valuable material for a similar study of personality types. These findings show that personality inference from EEG signals outperforms state-of-the-art clear behavioral indicators in classification accuracy.

### 4.2. Proposed DeepLSTM Model

Various algorithms for learning machines are used for the recognition and description of personality characteristics in literature. The DeepLSTM model for personality traits classification with the use of EEG signals is used in this work.

Figure 4 includes the architectures of the DeepLSTM cell network used for classifying the personality traits by using EEG signals in this analysis. The DeepLSTM network has been established on the backend in Python 3.6 Keras 2.0.9 on TensorFlow 1.4.0.

In DeepLSTM architecture, there are 3 LSTM layers, with 512 memory units in the first layer, 256 memory units in the second layer, and 128 memory units in the third layer. In all proposed architectures, the dropout layer is also used, and the probability value is 0.2. In the model between existing layers, the dropout layer is applied to previous layer outputs, which are fed to the layer, as shown in Figure 4. A layer's outputs are arbitrarily subsampled under dropout layer. The memorization capability of the DeepLSTM model is due to the dropout regularization [28]. Furthermore, the model is trained faster with the 0.2 dropouts, overfitting is reduced, and the proposed DeepLSTM model performs better in terms of prediction. The “tanh” function is used as an activation function and generates the output of 64 units.

(1) $$\begin{array}{c} \tanh\left(x\right)=\frac{2}{1+e^{-2x}}-1. \end{array}$$

“Softmax” is used as an activation function in the last layer and 4 outputs are generated representing four personality classes. The key benefit of using the softmax as an activation function is the range of output probabilities, which will be between 0 and 1. It returns each class's probabilities, with the target class having the highest probability.

(2) $$\begin{array}{c} \text{Softmax}\left(x_{i}\right)=\frac{\exp\left(x_{i}\right)}{\sum_{j}\exp\left(x_{j}\right)}. \end{array}$$

LSTM cells and dropout layers are utilised to discover the role of EEG signals. The overfitting of these systems was minimized by restricting unit coadapting in the dropout layer of our DeepLSTM architectures. The dense layer, the loss function for these network architectures, is categorical cross-entropy and the batch size is 40. The adaptive moment estimation optimizer (Adam) is used for a learning rate of 0.001. The normalization is applied to the dataset input features with the MinMaxScaler function after loading the dataset. This function normalizes each feature because of which each feature contributes in a maintained manner. It decreases the internal covariate transition, resulting in a change in network activation distribution due to shifts in network parameters during training. The normalization of the proposed network enhances training, reducing the change in the internal covariance. It also helped improve the optimization phase by stopping weights from bursting around the entire site by limiting them to a specific set. An undesired advantage of normalization is that it often allows the mechanism to regularize somewhat. In the parameter specified by Table 2, the proposed DeepLSTM network is initialized [29]. We test the output of our proposed DeepLSTM model, which classifies EEG signals as an output value into five personality groups, for 500 epochs with a batch size of 40. The DeepLSTM model was evaluated using the suggested EEG dataset as well as the publicly available ASCERTAIN EEG dataset.

The article "EEG-Based Personality Prediction Using Fast Fourier Transform and DeepLSTM Model" was published in 2021. Journal: Comput Intell Neurosci.

The proposed architectures and parameters were chosen based on our own experiments with nearby architectures (in terms of layers and nodes). In terms of accuracy, the proposed DeepLSTM architecture outperforms their nearby architecture.

## 5. Experimental Results

The results of the DeepLSTM model for classifying the EEG signals and to check our system's efficacy are presented next. The computer environment is composed of 3.4 GHz devoted to the 32 GB RAM-based Python (3.6) to incorporate DeepLSTM cell architecture and other states of the art, i.e., ANN, KNN, LibSVM, and HGP. The parameter values of the ANN, KNN, LibSVM, and HGP are the same as in [19, 30], respectively. The parameter values taken for the implementation of the DeepLSTM model are given in Table 2.

The dataset is typically split into two distinct sets, i.e., training sets and test sets. A general review of our method is carried out in this research of personality trait classification using EEG signals. We have separated the dataset into different training and testing partitions to equate them with existing literature. The performance assessment is conducted using a 50–50, 60–40, 70–30, and 10-fold partition scheme.

The article "EEG-Based Personality Prediction Using Fast Fourier Transform and DeepLSTM Model" was published in 2021. Journal: Comput Intell Neurosci.

In 50–50, 60–40, and 70–30 training-testing partition, 50%, 60%, and 70%, respectively, data is used for training, and 50%, 40%, and 30%, respectively, of the data is used for testing. The complete dataset is partitioned into approximately ten equal size blocks in a 10-fold cross-validation scheme; 90% of the dataset, i.e., nine blocks, becomes our training data, and 10% of the dataset, i.e. one block, becomes our testing data. This process is repeated ten times, with each time a different data block being used for testing. Also, our proposed model's sensitivity, precision, and specificity value for the 50–50, 60–40, 70–30, and 10-fold partition schemes are calculated.

### 5.1. DeepLSTM Architecture Evaluation

This study uses a deep learning algorithm to distinguish personality traits from EEG signals. In practice, the DeepLSTM model outperforms traditional machine learning algorithms because it has the capability of remembering the long-term dependence of sequential data in time, increasing the likelihood of correctness in a short period of time [31].

Table 3 represents the classification accuracy comparison for personality prediction DeepLSTM model on the ASCERTAIN and the proposed EEG datasets. For the ASCERTAIN and the proposed EEG datasets, the proposed DeepLSTM model maximum, average, and minimum classification accuracy for 50–50, 60–40, 70–30, and 10-fold cross-validation partition scheme is calculated.

The maximum classification accuracy of the proposed DeepLSTM model for 50–50, 60–40, 70–30, and 10-fold cross-validation partition scheme on the ASCERTAIN EEG dataset is 82.48%, 88.14%, 92.86%, and 95.32%, respectively.

The maximum classification accuracy of the proposed DeepLSTM model for 50–50, 60–40, 70–30, and 10-fold cross-validation partition scheme on the proposed EEG dataset is 84.56%, 91.52%, 94.82%, and 96.94%, respectively. From the results, it can be seen that the DeepLSTM model performs better in terms of performance on the ASCERTAIN and the proposed EEG datasets, and the classification accuracy of the DeepLSTM model is higher on our proposed EEG dataset than the ASCERTAIN dataset.

## 6. Discussion

This section discusses how the proposed deep learning-based DeepLSTM model works compared to conventional machine learning algorithms.

A comparison with standard conventional classification algorithms is carried out using the same collection of features as used in DeepLSTM-based methodology to show the advantages of incorporating deep learning into the classification of personality traits.

The KNN, ANN, LibSVM, and HGP are the other state-of-the-art approaches used for comparison. The classification accuracy comparison of personality traits is contained in Table 4. It contains the maximum, average, and minimum accuracy for the 50–50, 60–40, 70–30, and 10-fold partition schemes. The parameters and settings for these variables have all been implemented using the same technique to ensure that the findings and comparisons offered are unambiguous and consistent.

The article "EEG-Based Personality Prediction Using Fast Fourier Transform and DeepLSTM Model" was published in 2021. Journal: Comput Intell Neurosci.

The proposed deep learning approach has a greater impact than traditional machine learning algorithms. The DeepLSTM classification improved dramatically in classification accuracy, as per the results. Besides the rise in classification accuracy, the DeepLSTM classifier can also retain specificity greater than 92.86% on the ASCERTAIN dataset and 93.84% on the proposed EEG dataset, resulting in very low false prediction % rates. The sensitivity value of the DeepLSTM model for the ASCERTAIN dataset is 94.72%, and the proposed EEG dataset is 95.86% and is high in the other state-of-the-art methods, which shows that the DeepLSTM model correctly classifies the minority class samples. The precision value of the DeepLSTM model for the ASCERTAIN dataset is 93.48%, and the proposed EEG dataset is 94.44% and is high in the other state-of-the-art methods. The *F*1 score value of the DeepLSTM model for the ASCERTAIN dataset is 93.68%, and the proposed EEG dataset is 94.96% and is high in the other state-of-the-art methods.  Table 5 shows the relation of sensitivity, precision, specificity, and F1 score values of DeepLSTM for 50–50, 60–40, 70–30, and 10-fold data partitioning scheme.

Table 6 shows the statistical result disparity is illustrated by the two-tailed Mann–Whitney test [32]. The Mann–Whitney test is used to compute the *p* value relation in classification accuracy. The outcomes do not change significantly if the *p* value is greater than 0.05, and it is highly significant if the *p* value is less than 0.001. It is evident from the interventions in Table 6 that the solution provided by our proposed DeepLSTM model is statistically different from ANN, KNN, LibSVM, and HGP for the 50–50, 60–40, 70–30, and 10-fold data partitioning scheme. When the *p* values are contrasted with DeepLSTM for these classifiers, there is a significant variation in outcomes. The evaluation results suggest that the proposed DeepLSTM-based deep learning model for classifying personality traits provides accurate classification results.

## 7. Conclusion

During this study, we propose EEG signals-based personality prediction system using DeepLSTM-based deep learning model.

A new EEG dataset was also created using 40 film clips of Hindi and English languages. The proposed DeepLSTM model was also applied to the publicly available EEG dataset known as ASCERTAIN. Multiple experiments have been carried out to validate our results, which are helpful to compare our DeepLSTM model with existing methods. Fifty participants were involved and saw a few movie clips targeting eight different personality traits. This method uses NeuroSky MindWave mobile 2 to capture brain signals. Better results of sensitivity, precision, and specificity indicate that our approach beats the current literature. The classification accuracy of the proposed DeepLSTM model on our proposed EEG dataset is 96.94% for the 10-fold partition scheme and outperforms the results of the DeepLSTM model on the ASCERTAIN dataset having classification accuracy of 95.32%.

The article "EEG-Based Personality Prediction Using Fast Fourier Transform and DeepLSTM Model" was published in 2021. Journal: Comput Intell Neurosci.

We are currently using a single-channel device, and in the future, we will extend it to multichannel devices.

## Figures and Tables

**Figure 1:** Brainwave frequency bands.

**Figure 2:** Single-channel NeuroSky MindWave mobile 2.

**Figure 3:** Personality prediction framework using EEG signals and DeepLSTM model.

**Figure 4:** DeepLSTM cells network architecture.

**Table 1:** Sample of stimuli dataset clips to felicitate targeted personality traits for EEG data acquisition.

Personality trait	Film name	Length (minutes)	Clip content
Extrovert	IBIZA	2.8 min	Harper, an extrovert character exploring Spain
Introvert	Jab We Met	3.22 min	An introvert guy boards a random train where he meets a bubbly girl
Thinking	Slumdog Millionaire	2.6 min	An uneducated nobody from slums answers critical questions of knowledge to become a millionaire
Feeling	12 Years a Slave	3.61 min	An incredible true story of Solomon Northup, a free African-American, abducted and sold into slavery, fights not only to survive, but to retain his dignity
Sensing	URI: The Surgical Strike	2.88 min	The clip chronicles an event of the surgical strike lead by major for a covert operation against suspected militants
Intuitive	Confessions of a Shopaholic	3.5 min	An abstract and imaginative character, struggling with her enfeeble obsession with shopping
Judging	The Devil Wears Prada	2.9 min	A famed fashion designer life story of being systematic schedule which inspires both terror and a measure of awe.
Perceiving	3 Idiots	3.0 min	An aspiring engineering student delivers a life lesson in a very innovative manner

**Table 2:** DeepLSTM model formation parameter values.

Parameter	Value
Optimizer	Adam
Rate of learning	0.001
Rate of dropout	0.2
Loss function	Categorical cross-entropy
Metrics used	Accuracy
Size of batch	40

**Table 3:** Classification accuracy comparison for personality prediction of DeepLSTM model on the ASCERTAIN and proposed EEG datasets.

Dataset	Method	Validation technique	Accuracy		
			Max	Avg	Min
ASCERTAIN	DeepLSTM classifier	50–50	82.48	80.36	77.42
		60–40	88.14	85.63	81.46
		70–30	92.86	89.68	86.46
		10-fold	**95.32**	**94.16**	**91.98**

Proposed dataset	DeepLSTM classifier	50–50	84.56	82.44	79.62
		60–40	91.52	87.62	84.86
		70–30	94.82	91.68	88.72
		10-fold	**96.94**	**95.88**	**93.94**

Optimal values are represented in bold.

The article "EEG-Based Personality Prediction Using Fast Fourier Transform and DeepLSTM Model" was published in 2021. Journal: Comput Intell Neurosci.

**Table 4:** Classification accuracy comparison for personality prediction of DeepLSTM model with other state-of-the-art algorithms on the ASCERTAIN and the proposed EEG dataset.

Dataset	Method	Validation technique	Accuracy		
			Max	Avg	Min
ASCERTAIN	ANN	50–50	70.84	67.24	64.48
	KNN	50–50	67.64	64.26	62.23
	LIBSVM	50–50	77.28	73.84	71.86
	HGP	50–50	78.52	75.38	72.68
	DeepLSTM classifier	50–50	82.48	80.36	77.42

ASCERTAIN	ANN	60–40	74.34	69.86	67.74
	KNN	60–40	70.38	68.16	65.68
	LIBSVM	60–40	79.86	77.28	75.46
	HGP	60–40	81.27	78.73	76.08
	DeepLSTM classifier	60–40	88.14	85.63	81.46

ASCERTAIN	ANN	70–30	75.18	73.16	69.94
	KNN	70–30	72.82	70.84	68.62
	LIBSVM	70–30	83.26	81.62	79.86
	HGP	70–30	86.64	83.38	80.74
	DeepLSTM classifier	70–30	92.86	89.68	86.46

ASCERTAIN	ANN	10-fold	78.82	74.64	72.46
	KNN	10-fold	74.36	72.37	70.25
	LIBSVM	10-fold	84.82	82.42	80.28
	HGP	10-fold	86.12	83.86	81.84
	DeepLSTM classifier	10-fold	**95.32**	**94.16**	**91.98**

Proposed dataset	ANN	50–50	72.84	69.36	66.48
	KNN	50–50	69.32	66.92	63.86
	LIBSVM	50–50	79.74	76.64	73.86
	HGP	50–50	80.36	77.83	74.89
	DeepLSTM classifier	50–50	84.56	82.44	79.62

Proposed dataset	ANN	60–40	76.16	73.28	70.12
	KNN	60–40	72.64	70.62	68.54
	LIBSVM	60–40	81.26	79.58	77.82
	HGP	60–40	83.28	80.94	78.63
	DeepLSTM classifier	60–40	91.52	87.62	84.86

proposed dataset	ANN	70–30	78.62	73.94	71.28
	KNN	70–30	74.68	72.36	70.82
	LIBSVM	70–30	85.64	83.70	81.58
	HGP	70–30	87.69	84.74	82.84
	DeepLSTM classifier	70–30	94.82	91.68	88.72

Proposed dataset	ANN	10-fold	80.24	76.54	74.98
	KNN	10-fold	76.82	74.64	72.28
	LIBSVM	10-fold	88.04	85.16	83.26
	HGP	10-fold	90.32	86.93	84.78
	DeepLSTM classifier	10-fold	**96.94**	**95.88**	**93.94**

Optimal values are represented in bold.

**Table 5:** Comparison of sensitivity, precision, and specificity of DeepLSTM model for various partition schemes.

Dataset	Validation technique	Sensitivity (%)		Precision (%)		Specificity (%)		*F*1 score (%)	
		Mean ± Std		Mean ± Std		Mean ± Std		Mean ± Std	
ASCERTAIN	**50–50**	81.64	±3.08	80.53	±3.12	78.42	±2.84	80.56	±2.36
	**60–40**	87.76	±3.14	86.82	±3.24	85.94	±2.68	86.44	±2.44
	**70–30**	91.49	±3.16	90.56	±3.42	89.67	±2.36	90.40	±3.42
	**10-fold**	**94.72**	± **3.16**	**93.48**	± **3.12**	**92.86**	± **2.98**	**93.68**	± **2.84**

Proposed dataset	**50–50**	83.46	±3.14	82.75	±3.15	81.14	±3.24	82.46	±3.18
	**60–40**	90.74	±3.24	89.25	±3.16	88.94	±3.18	89.46	±3.32
	**70–30**	93.54	±3.14	92.85	±3.25	91.94	±3.42	92.28	±3.24
	**10-fold**	**95.86**	± **3.18**	**94.44**	± **3.14**	**93.84**	± **3.12**	**94.96**	± **3.16**

Optimal values are represented in bold.

The article "EEG-Based Personality Prediction Using Fast Fourier Transform and DeepLSTM Model" was published in 2021. Journal: Comput Intell Neurosci.

**Table 6:** *p* value comparison for DeepLSTM using Mann–Whitney test.

	Training-testing	ANN				KNN				LibSVM				HGP			
	Partition	*p* value		Significance		*p*-value		Significance		*p* value		Significance		*p* value		Significance	
DeepLSTM	50–50	2.681 x	10^−11^	Highly	Significant	1.450 x	10^−11^	Highly	Significant	1.9543	10^−11^	Highly	Significant	1.8563	10^−11^	Highly	Significant
	60–40	2.634 x	10^−11^	Highly	Significant	1.350 x	10^−11^	Highly	Significant	1.8703	10^−11^	Highly	Significant	1.8363	10^−11^	Highly	Significant
	70–30	2.576 x	10^−11^	Highly	Significant	1.270 x	10^−11^	Highly	Significant	1.8423	10^−11^	Highly	Significant	1.7946	10^−11^	Highly	Significant
	10-fold	2.486 x	10^−11^	Highly	Significant	1.235 x	10^−11^	Highly	Significant	1.7856	10^−11^	Highly	Significant	1.7637	10^−11^	Highly	Significant

Optimal values are represented in bold.

## Data Availability

The data are available on request from the corresponding author.
